# Endovascular Treatment of Internal Iliac Artery Stenosis in Patients with Buttock Claudication

**DOI:** 10.1371/journal.pone.0073331

**Published:** 2013-08-08

**Authors:** Jip F. Prince, Maarten L. J. Smits, Joost A. van Herwaarden, Mark J. Arntz, Evert-Jan P. A. Vonken, Maurice A. A. J. van den Bosch, Gert Jan de Borst

**Affiliations:** 1 Department of Radiology, University Medical Center Utrecht, Utrecht, the Netherlands; 2 Department of Vascular Surgery, University Medical Center Utrecht, Utrecht, the Netherlands; Villa Torri Hospital, Italy

## Abstract

**Aim:**

To assess the technical feasibility and clinical outcome of percutaneous transluminal angioplasty (PTA) with and without stent placement for treatment of buttock claudication caused by internal iliac artery (IIA) stenosis.

**Methods:**

Between September 2001 and July 2011, thirty-four patients with buttock claudication underwent endovascular treatment. After angiographic lesion evaluation PTA with or without stent placement was performed. Technical success was recorded. Clinical outcome post-treatment was assessed at three months post-intervention and was classified as: 1) complete relief of symptoms, 2) partial relief, or 3) no relief of symptoms. Complications during follow-up were recorded.

**Results:**

Forty-four lesions in 34 symptomatic patients were treated with PTA. Eight lesions were treated with additional stent placement. Technical success was achieved in 40/44 lesions (91%). Three procedure-related minor complications occurred, i.e. asymptomatic conservatively treated intimal dissections. After a median of 2.9 months, patients experienced no relief of symptoms in 7/34 cases (21%), partial relief in 14/34 cases (41%), and complete relief in 13/34 cases (38%). Six patients required a reintervention during follow-up.

**Conclusion:**

Endovascular treatment of IIA stenosis has a high technical success rate and a low complication rate. Complete or partial relief of symptoms is achieved in the majority (79%) of patients.

## Introduction

Internal iliac artery (IIA) stenosis may lead to symptoms including pain in the buttocks or hips, extending to the upper leg [1]. In males, impotence can be found. The pain can be difficult to differentiate from coxarthrosis or neurogenic claudication [2,3].

Upon clinical suspicion of IIA stenosis, an ankle brachial pressure index can be normal as this does not include, or may not optimally visualize, the whole IIA. Color flow duplex ultrasonography (DUS) and computed tomography angiography (CTA) and/or magnetic resonance angiography (MRA) can confirm the presence of an isolated IIA stenosis or a combined IIA stenosis with stenotic inflow of the common iliac artery [4].

Treatment options range from a) conservative management including exercise therapy, life-style changes, and antiplatelet therapy, to b) minimally invasive endovascular treatment, i.e. percutaneous transluminal angioplasty (PTA), with or without stent placement, supported by antiplatelet therapy [4–6].

There is scant literature on the technical efficacy and clinical outcome of endovascular treatment of IIA in patients with buttock claudication [7]. Furthermore, little data has been reported on the durability of symptom relief following endovascular treatment.

In this study the technical feasibility, safety, and three months clinical outcome with mid-term patency rates of endovascular treatment, including PTA with or without stent placement, were assessed in patients with buttock claudication due to angiographically confirmed significant internal iliac artery stenosis.

##  Materials and Methods

### Definition of buttock claudication

Symptomatic buttock claudication was defined as a composite of two findings. First, the presence of invalidating and intermittent pain and/or weakness in the buttock or thigh related to walking/exercise, as reported by the patient. Second, the finding of a significant stenosis in the IIA on the symptomatic side, defined as a reduction of more than 50% of the vessel diameter, as found on digital subtraction angiography (DSA).

### Patient selection

Between September 2001 and July 2011, all consecutive patients undergoing endovascular treatment for buttock claudication due to IIA stenosis with or without concomitant inflow stenosis in the common iliac artery (CIA) were included. Patients without concomitant lesions were analyzed separately to prevent confounding. Patients with IIA occlusion were not considered appropriate candidates for revascularization and were excluded from the present analysis. All baseline characteristics, data of the endovascular procedure (including treatment of concomitant lesions) and follow-up were retrospectively collected from the medical records.

### Ethics statement

The institutional review board of the University Medical Center Utrecht (Utrecht, the Netherlands) approved this retrospective case cohort study and issued a waiver for patient informed consent.

### Clinical workup

Patients with complaints of buttock claudication were seen by a vascular surgeon. Neurologic and orthopedic causes were excluded based on anamnesis and physical examination if possible, or referred to the relevant specialist. Upon suspicion of a lesion in the iliac arteries, DUS, CTA, or MRI was performed. If an arterial iliac lesion was shown, the treatment indication was confirmed in a multidisciplinary vascular meeting with vascular surgeons and interventional radiologists present. A DSA was then performed, of which details can be found below.

### Treatment

All patients were referred to the cathlab for endovascular treatment. Patients were treated by an experienced interventional radiologist.

Following subcutaneous injection of 1% xylocaine, a sheath was introduced in the ipsi- or contralateral femoral artery. The brachial artery was used if access using the iliac vessels was not feasible, e.g. due to a steep angle of both CIAs with the abdominal aorta. In total, 2500 units of heparin were administered. When the femoral artery was punctured, a 6 French (F) sheath was placed over the aortic bifurcation. The stenosis was confirmed on DSA using Visipaque 270 contrast (GE Healthcare, Little Chalfont, UK). If necessary, additional oblique projections were made and vessel sizes were measured. The grade of stenosis was assessed.

If the IIA stenosis was accompanied by a significant stenosis (>50%) in the external iliac artery (EIA) or CIA, additional lesions were treated by either PTA or stent placement. An angled guide wire was used to pass the stenosis, followed by placement of a balloon catheter. The balloon was inflated to nominal pressure using a calibrated inflation device for two minutes (Basix Compak, Merit Medical, Galway, Ireland). After treatment, the response was evaluated on DSA. If PTA was unsuccessful (i.e. the angiographically assessed stenosis grade remained ≥30%), additional placement of a balloon-expendable metal stent (Palmaz Blue, Cordis) was considered.

Clinical follow-up consisted of a visit to the outpatient department 3 months after treatment. Patients were discharged from outpatient control if they were symptom-free or with sufficient symptom relieve, and were requested to return if symptoms re-occurred.

### End point definition

The primary endpoint of our study was severity of buttock claudication three months post procedure as compared to the prior situation. This comparison was quantified in three categories: 1) complete relief of symptoms, 2) partial relief, or 3) no relief of symptoms. Patients’ complaints were subjectively assessed by a vascular surgeon with regard to buttock pain free walking distance, intensity of pain during exercise, and rest pain. Secondary endpoints were technical success, defined as angiographic residual lumen stenosis <30%, periprocedural complications, the need to perform reintervention, and occurrence of occlusion during follow up. To exclude confounding by concomitant lesions, the subgroup of patients with treatment of only IIA stenosis was also assessed separately.

### Statistical analysis

Patency of treated vessels was expressed as primary and secondary patency rate.

Primary patency was defined as uninterrupted patency with no additional procedure performed. Secondary patency was defined as if patency was restored by an additional intervention (in accordance with published guidelines) [8].

The timing of angiographic confirmation of patency loss was used for patency rate calculations with Kaplan-Meier method. A cut-off of 10% of standard error of patency rate estimate was applied.

All risk factors and treatment characteristics were univariately analyzed for prediction of a favorable treatment response. Clinical outcome was dichotomized in patients with none to partial relief of complaints, and patients with complete relief of symptoms. Variable were analyzed using a two-tailed Fisher’s exact test and p-values were calculated. A p-value smaller than 0.05 was considered statistically significant. Analyses were performed using SPSS, version 15 (IBM, North America, New York, NY, USA).

## Results

### Patients

A total of 44 stenotic IIA lesions in 34 patients were treated. Of these patients, 31 were male. The median age was 67 years (range 52-83 years). Some patients experienced bilateral buttock claudication (16/34, 47%), others only on the right (9/34, 26%) of left side (9/34, 26%). Most patients had earlier treatment for PAD (n=29), hypercholesterolemia (n=29), or hypertension (n=27). Further baseline characteristics and the presence of other risk factors are presented in Table 1.

**Table 1:** Baseline characteristics.

**Characteristic**		**Number (percentage) or median (range)**
Gender	Male	31 (91%)
	Female	3 (9%)
Age (*years*)		67 (52-83)
Fontaine classification^a^	1	0 (0%)
	2a	12 (35%)
	2b	19 (56%)
	3	2 (6%)
	4	1 (3%)
Side of buttock complaints	Left	9 (26%)
	Right	9 (26%)
	Both	16 (47%)
ABI of treated limb		0.96 (0.39-1.51)
Risk Factors^b^	Smoking	12
	Overweight (BMI >25)	20
	Diabetes	14
	Hypertension	27
	Hypercholesterolemia	29
	Familial risk factors	15
	Earlier invasive treatment for PAD	29
	Impotence	3

^a^ of lower extremity

^b^ if reported in medical records, as such, no percentage calculation was possible

ABI = ankle brachial pressure indexPAD = Peripheral artery disease

Percentages might not add up to 100% due to rounding

### Lesions

After pre-procedural workup using DUS, CTA, or MRA, a DSA showed 35/44 lesions (80%) in the IIA origin, and 9/44 (20%) more distal IIA lesions. A concomitant lesion of the contralateral IIA (stenosis or occlusion) was present in 15/34 (44%) patients, of which 7 experienced bilateral complaints. An ipsilateral CIA stenosis was present in 6/34 (18%) of the patients.

### Treatment

Percutaneous transluminal angioplasty of the IIA stenosis was performed in all patients. The mean balloon diameter used was 5mm (range 3-7mm). In eight patients, the stenosis was not sufficiently relieved, or relapsed, and a balloon-expandable bare-metal stent (5-8mm in diameter) was placed in the IIA in addition to the PTA. The ipsilateral CIA was treated in 5/44 (11%) of the lesions. A bilateral treatment of both IIAs was performed in 10/34 (29%) patients. Treatment characteristics are summarized in Table 2 and the inclusion, treatment, and results are displayed in Figure 1. Technical success was achieved in 40 out of 44 (91%) lesions (Figure 2). In four patients >30% stenosis remained after endovascular treatment.

**Table 2:** Diagnosis, treatment and clinical outcome.

**Characteristic**		**Number (%)**
Diagnosis	Lesions / Patients	44/34
	Contralateral IIA occlusions	4/34 (12%)
	Contralateral IIA or CIA stenosis	15/34 (44%)
	Ipsilateral CIA stenosis	6/34 (18%)
	Bilateral IIA stenosis or occlusion	15/34 (44%)
	Origin stenosis	35/44 (80%)
	Stent CIA or EIA causing stenosis	5/44 (11%)
*Treatment*	Access via femoral artery	30/34 (88%)
	Access via brachial artery	4/34 (12%)
	Size balloon PTA (3mm-4-5-6-7)	7-11-8-16-2
	Stents placed	8/34 (24%)
	Isolated IIA treatment	22/34 (65%)
	Bilateral IIA treatment	10/34 (29%)
	CIA treatment ipsilateral	5/44 (11%)
	Technical success	40/44 (91%)
	Complications	3/34 (9%)
*Clinical Outcome After 3 Months (total of 34 patients)*	Group 1 (no relief)	7 (21%)
	Group 2 (partial relief)	14 (41%)
	Group 3 (total relief)	13 (38%)
*Clinical Outcome After 3 Months for patients with isolated IIA treatment (total of 22 patients)*	Group 1 (no relief)	5 (23%)
	Group 2 (partial relief)	8 (36%)
	Group 3 (total relief)	9 (41%)

*CIA* = Common iliac artery*EIA* = External iliac artery*IIA* = Internal iliac artery*PTA* = Percutaneous transluminal angioplasty

**Figure 1:** Flowchart of study design. IIA = Internal Iliac Artery. CIA = Common Iliac Artery. EIA = External Iliac Artery.

**Figure 2:** Treatment of a patient. (a) Digital subtraction angiography of the left common iliac artery showing a proximal stenosis of the internal iliac artery (IIA), with sub-optimal filling of subsequent branches. (b) Result after treatment with 5 and 6 mm percutaneous transluminal angioplasty, showing residual origin stenosis of the IIA of more than 30%. (c) Subsequent stent placement (Palmaz 6 mm diameter) reduced the stenosis grade to less than 30%, and provided adequate distal blood flow. (d) Overlay of Figure c showing branches of mentioned vessels, guide wire position (white dotted line) and placed stent (white mesh). CIA = Common Iliac Artery. EIA = External Iliac Artery. IIA = Internal Iliac Artery.

### Complications

Procedural related complications occurred in 3/34 patients (9%). In one patient, a small dissection developed in the ipsilateral CIA during treatment. The second patient underwent treatment for both the IIA and the EIA. In the EIA, a small dissection was caused at the bifurcation. Blood flow was not compromised in both cases and both dissections were conservatively treated. The third complication occurred upon passing the stenosis in the left IIA. A dissection was caused, which obstructed the vessel lumen. The contralateral IIA stenosis was successfully treated. During follow-up, the patient reported neither deterioration nor improvement of complaints.

### Primary endpoint: follow up at three months

After a median of three months, 7/34 (21%) patients reported no symptomatic relief. One patient was diagnosed with coxarthrosis shortly after IIA treatment. On the other hand, 14/34 (41%) patients experienced a significant improvement while 13/34 (38%) patients had a complete relief of symptoms.

Of all patients treated, 22 patients received treatment for solely their IIA lesion, and no other inflow arteries. In this subgroup, 30 lesions were treated. After a median of 2.9 months, 5/22 (23%) patients did not experience symptomatic relief. A total of 8/22 (36%) patients experienced partial improvement, and in 9/22 (41%) patients the buttock claudication disappeared completely.

### Follow up

After a median follow up of 10 months (range 1-116 months) in the full cohort of 34 patients, three patients presented with ipsilateral occlusion of the iliac tract (3/34, 9%). One patient developed an occlusion in the CIA extending into the IIA, 12 months after initial treatment. This patient successfully received thrombolytic treatment and additional stent placement in the EIA for signs of a dissection. Another patient developed an EIA occlusion distal of a prior placed CIA stent, 8 months after treatment. The IIA was patent. This patient received urokinase treatment with good effect, and antithrombotic therapy consisting of acenocoumarol was added to her antiplatelet therapy. A third patient had an occlusion of the treated IIA, discovered 68 months after PTA treatment. Since there were no complaints precipitating the occlusions, no time of occlusion could be determined and it was decided not to treat.

Another 6/34 (18%) patients required reinterventions due to progressive symptomatic restenosis at the site of the initial target lesion, which, in all cases, occurred more than 4 months after primary treatment. Two patients underwent re-PTA and in four patients five additional stents were placed (Table 3).

**Table 3:** Follow up.

**Characteristic**	**Number (%) or median (range)**
Follow up (*months*)	10 (1-116)
Iliac occlusions	3 (9%)
Reinterventions	6 (18%)
Additional stent placement (*patients*)	5 (15%)
Deaths^a^	3 (9%)
Loss to follow-up^b^	0 (0%)

^a^ None were related to IIA treatment

^b^ If no information of first visit after procedure could be obtained

No treatment related deaths were noted during follow-up. Three patients died during follow-up. The death of one patient was related to a Merkel cell carcinoma, and occurred 53 months after endovascular treatment. The other patient died due to complications of abdominal surgery, 23 months after treatment. The third patient died 15 months after treatment due to an intracerebral hemorrhage.

### Patency rates

The primary patency rate after 7.8 months was 77% (standard error 9.0%). The median survival time was 30 ± 12.3 months. Since there was only one occlusion in the IIA, which was untreated for reasons mentioned above, the secondary patency rate had one endpoint, and the standard error exceeded 10% for all values.

The analysis of risk factors and variables of diagnosis and treatment did not show any particular feature which was significantly associated with a favourable outcome.

## Discussion

Only a few studies with limited number of patients assessed the clinical outcome of endovascular treatment of patients with buttock claudication due to internal iliac artery stenosis (see Table 4) [7]. In our single center experience, endovascular treatment of IIA stenosis showed a high technical success rate. PTA of the IIA, with or without stent implantation, seems therefore feasible and safe, with no major complications and acceptable rate of minor complications. After three months, the majority of patients had (partial or complete) relief of clinical symptoms. During further follow up the mid-term patency rate is high.

**Table 4:** Review of literature concerning endovascular therapy for IIA stenosis or occlusion.

**Study**	**Type of IIA lesions treated**	**Exclusion of neurologic of orthopedic causes**	**n (lesions /patients)**			**PTA**	**Stents placed^a^**	**Technical success**	**Complications**	**Complete relief^b^**	**Partial relief**		**No relief**
Morse et al. (1986)[11]	stenosis^c^	not mentioned	2	/	2	2	0	100%	0%	1 (50%)	1 (50%)		0 (0%)
Smith et al. (1992)[3]	stenosis^c^	not mentioned	2	/	2	2	0	100%	0%	1 (50%)	1 (50%)		0 (0%)
Batt et al. (2006)[6]	stenosis or occlusion of SGA^c^	physical examination	7	/	6	7	0	100%	0%	5 (83%)	1 (17%)^d^		
Huetink et al. (2008)[1]	stenosis^c^	excluded, not mentioned how	4	/	3	4	0	100%	0%	2 (67%)	1 (33%)	0 (0%)	
Adlakha et al. (2009)[12]	occlusion	not mentioned	2	/	2	2	2	100%	0%	2 (100%)	0 (0%)	0 (0%)	
Donas et al. (2009)[7]	stenosis or occlusion^c^	clinical evaluation + CT-scan	22	/	21	14	8	100%	0%	21 (100%)	0 (0%)	0 (0%)	
Thompson et al. (2009)[9]	stenosis or occlusion^c^	not mentioned	15	/	9	7	8	100%	0%	7 (78%)	0 (0%)	2 (22%)	
Prince et al. (2013)^e^	>50% lumen obstruction	physical examination	44	/	34	36	8	91%	9%	13 (38%)	14 (41%)	7 (21%)	

*IIA* = Internal iliac artery*PTA* = Percutaneous transluminal angioplasty*SGA* = superior gluteal artery

^a^ Number of stents placed in the IIA or distal arteries, treatment was sometimes accompanied by PTA

^b^ Treatment results were classified as complete, partial or no relief based on description in article

^c^ Minimum stenosis grade not mentioned

^d^ Partial or no relief

^e^ This study

Buttock claudication as a diagnosis may have a vascular origin, but symptoms may also be mimicked by other disease entities such as coxarthrosis and neurogenic claudication, which therefore should be in the differential diagnosis at baseline [3]. Prior studies used different methods of excluding neurogenic or orthopedic causes, as seen in Table 4. However, in a patient with symptoms which are relieved after a resting period and who has a proven significant IIA stenosis our results indicate that this patient can be offered endovascular treatment with a low threshold.

In reviewing the outcomes after IIA PTA/selective stenting we also performed an analysis including only patients who were treated for isolated IIA lesions (and absence of concomitant common iliac lesions). Severe stenotic IIA lesions are often accompanied by concomitant stenoses in the CIA or EIA. Treating the proximal artery (CIA) can have beneficial effects on patient outcome by itself. When a stenosis in the IIA extends in the EIA, and both significantly comprise the flow, a combined treatment will be necessary (see Figure 3). Simultaneous treatments will affect treatment outcome. The outcome of treating solely the IIA lesion will provide more insight. However, within the present series, the outcome of this subgroup did not differ from the outcome of the full cohort.

**Figure 3:** Treatment of a patient (#7) with bilateral buttock claudication and iliac stenoses. (a) Digital subtraction angiography showing the sheath retrogradely advanced to the common iliac artery. Stenoses of the external and internal iliac arteries are visible at their respective origins (arrows). (b) Results of percutaneous transluminal angioplasty of the external iliac artery with a 7 mm balloon and the internal iliac artery with a 4 mm balloon catheter. CIA = Common Iliac Artery. EIA = External Iliac Artery. IIA = Internal Iliac Artery.

During treatment of 44 lesions in 34 patients, three complications occurred (i.e. two dissections, one occlusion). Upon further follow up, no clinically relevant sequelae were found in any patient. This complication rate is comparable with other retrospective cohort studies in the literature [6,7,9].

PTA therapy (with or without stent) for IIA claudication yielded a partial to full relief of complaints in 92% of patients. The outcome of our treatment was evaluated after three months by a subjective outcome measure, the complaints reported by the patient as interpreted by the vascular surgeon. This is a limitation, as imaging or transcutaneous oxygen tension (TcPO2) can provide more objective measures. Furthermore, it is difficult to quantify patients’ complaints, so a distinction was made between full, partial or no relief. Quantification could have been done more thoroughly using standardized questionnaires. However, relevant literature often describes outcome as successful or not. This study provides a more quantified and clinically applicable outcome measure, as seen in Table 4.

If vessel patency decreases over time, PTA can be repeated. During follow up we performed reinterventions in four patients, all four because of residual complaints. Patency rates might be improved by placement of a stent [10]. Our limited number of primary stenting (n=5), stenting only when PTA was unsuccessful, and our retrospective study design did not allow us to analyze possible differences between patients receiving a stent and those who did not. Future prospective studies might consider IIA stenting as the primary treatment approach, or include a double treatment arm comparing primary PTA with primary stenting.

Another limitation of this study is the lack of structural follow-up, due to the retrospective study design. It also means that, due to lack of data, some determinants, such as impotency, cannot be evaluated for their association with the patients’ outcome. Impotency is a complaint often accompanying buttock claudication [6]. This compromises the validity of clinical outcome, and makes that our conclusions can be stated for the three months period of follow-up only.

## Conclusion

Endovascular treatment of patients with buttock claudication due to internal iliac artery stenosis is safe and effective in symptom relief in the majority of patients at short-term follow-up. Longer term durability needs to be awaited.
